# Optimal Deep Learning Enabled Prostate Cancer Detection Using Microarray Gene Expression

**DOI:** 10.1155/2022/7364704

**Published:** 2022-03-10

**Authors:** Abdulrhman M. Alshareef, Raed Alsini, Mohammed Alsieni, Fadwa Alrowais, Radwa Marzouk, Ibrahim Abunadi, Nadhem Nemri

**Affiliations:** ^1^Department of Information Systems, Faculty of Computing and Information Technology, King Abdulaziz University, Jeddah, Saudi Arabia; ^2^Department of Pharmacology, Faculty of Medicine, King Abdulaziz University, Jeddah, Saudi Arabia; ^3^Department of Computer Sciences, College of Computer and Information Sciences, Princess Nourah bint Abdulrahman University, P. O. Box 84428, Riyadh 11671, Saudi Arabia; ^4^Department of Information Systems, College of Computer and Information Sciences, Princess Nourah bint Abdulrahman University, P.O. Box 84428, Riyadh 11671, Saudi Arabia; ^5^Department of Information Systems, College of Computer and Information Sciences, Prince Sultan University, P.O. Box No. 66833, Rafha Street, Riyadh 11586, Saudi Arabia; ^6^Department of Information Systems, College of Science and Arts at Muhayel, King Khalid University, Mahayel Aseer, Saudi Arabia

## Abstract

Prostate cancer is the main cause of death over the globe. Earlier detection and classification of cancer is highly important to improve patient health. Previous studies utilized statistical and machine learning (ML) techniques for prostate cancer detection. However, several challenges that exist in the investigation process are the existence of high dimensionality data and less number of training samples. Metaheuristic algorithms can be used to resolve the curse of dimensionality and improve the detection rate of artificial intelligence (AI) techniques. With this motivation, this article develops an artificial intelligence based feature selection with deep learning model for prostate cancer detection (AIFSDL-PCD) using microarray gene expression data. The AIFSDL-PCD technique involves preprocessing to enhance the input data quality. In addition, a chaotic invasive weed optimization (CIWO) based feature selection (FS) technique for choosing an optimal subset of features shows the novelty of the work. Moreover, the deep neural network (DNN) model can be applied as a classification model to detect the existence of prostate cancer in the microarray gene expression data. Furthermore, the hyperparameters of the DNN model can be effectively adjusted by the use of RMSprop optimizer. The design of CIWO based FS technique helps for reducing the computational complexity and improve the classification accuracy. The experimental results highlighted the betterment of the AIFSDL-PCD approach on the other techniques with respect to distinct measures.

## 1. Introduction

In recent times, cancer is the leading cause of death worldwide. Generally, around 1 death from 6 overall deaths is because of cancer [1]. Therefore, in 2030, several new cases predicted annually might increase up to 25 million [2]. But early diagnoses of cancer might save billions of dollars and countless lives. The earlier prediction and identification of cancer is very crucial for cancer research and patient health. Once cancer is detected at earlier stages, treatment is highly efficient. In the past, classification of cancer is based on clinical and morphological technologies [3]. The innovative technologies have made considerable development in precise observation of hundreds of cancer genes via gene expression data. This method provides a massive amount of information to the authors for exploring several knowledge; however it has certain problems [4]. The key challenges of microarray data are low sample size and high dimensionality. Additionally, many microarray cancer information is noisy and could not be extremely helpful in the diagnosis of cancer [5]. Nowadays, categorizing cancer type more accurately and precisely and selecting most important genes associated with the cancer is one of the key challenges in the study [6].

Prostate cancer (PCa) is the 3rd one of the general detected cancers around the world, after breast and lung cancer, and the 5th cause of cancer-specific deaths in males [7]. In the past decades, researchers focus more on the prediction, diagnosis, and prognosis of PCa results taking the next step with help of Statistics and Artificial Intelligence (AI) technology. The usage of computer-based learning methods developed a significant research field in PCa. Generally, gene expression data contains large amount of genes; some authors evaluated and analyzed the cancer classification problems by utilizing different machine learning (DL), data mining (DM), and statistical based algorithms [8]. Several ML methods have attained lot of success better and classification performance in the cancer classification [9]. But, still, there are few problems with this approach which makes the cancer classification nontrivial tasks [10]. A disadvantage of conventional ML approach is needing preengineered organization of new input data as to structured data sets. The DL approach is a field of ML that employed layered structure for building sophisticated modules with the capacity to understand complex information [11]. This capability allows DL algorithms to demonstrate conventional ML techniques from multiple domains such as speech recognition computer vision, image classification, and so on.

The gene expression data comprises many redundant, noisy, and irrelevant items. The informative ratio to noisy data is 1 : 10 which degrade the performances of clustering when traditional approaches are employed directly to the comprehensive feature set. Hence, the informative feature selection (FS) technique plays an important role in higher-dimension gene expression data for biological data retrieval [12]. The FS method is separated into two classes. The initial class includes semisupervised, supervised, and unsupervised methods based on availability of historical data. The next class comprises ensemble, filter, wrapper, embedded, and hybrid approaches based on how they concatenate the selection by modeling. Each of these approaches has its disadvantages and advantages. In general, the hybrid approach is superior to the wrapper methods since it is less prone to overfitting. But the ensemble methodology is very flexible and robust [13]. The large dimension of gene expression data includes irrelevant, noise, and redundant items which makes it hard to examine. In this study, the FS methods are employed to lower the dimension of information for analysis of gene expression. Previously, the evolutionary learning method has been used effectively in distinct microarray researches, for example, to select informative subset of genes, for biclustering and sample, and clustering classification.

This article develops an artificial intelligence based feature selection with deep learning model for prostate cancer detection (AIFSDL-PCD) using microarray gene expression data. The AIFSDL-PCD technique derives a chaotic invasive weed optimization (CIWO) based FS technique for choosing an optimal subset of features. In addition, the deep neural network (DNN) model can be applied to prostate cancer classification utilizing the microarray gene expression data. Besides, the hyperparameters of the DNN model can be effectively adjusted by the use of RMSprop optimizer. For examining the betterment of the AIFSDL-PCD technique, a comprehensive experimental analysis is carried out and the results are examined under several aspects.

The rest of the study is planned as follows.  Section 2 offers the literature review, Section 3 presents the proposed model, Section 4 elaborates the performance validation, and Section 5 draws the conclusion.

## 2. Literature Review

Tavasoli et al. [14] presented a classification technique which employed metaheuristic and SVM algorithms. The optimization of the SVM hyperparameters for the RBF is implemented by utilizing the modified Water Cycle Algorithm (mWCA). The result indicates that the ensemble performance of gene-mWCA SVM (EGmWS) was regarded as effective methodology compared to related methodologies in terms of accuracy and solving the uncertainty problems. Elmarakeby et al. [15] designed a P-NET—a biologically informed DL method—for stratifying patients with PCa by treatment resistance state and gauging molecular driver of treatment resistance to therapeutic target via method interpretability. They demonstrated that P-NET could forecast cancer state by utilizing molecular information with performances, i.e., better than other modeling techniques.

Glaab et al. [16] estimated a rule-based evolutionary ML method, GAssist, and BioHEL, on three public microarray cancer data sets, attaining simple rule-based model for sample classifier. Compared to other standards of microarray, sample classification depends on three different FS methods. Darendeli et al. [17] focused on providing different perspectives of cancer diagnoses with DL method on gene expression data. In this work, RNA-Seq data of around thirty distinct kinds of cancer patients and the normal tissue RNA-Seq data from GTEx and Cancer Genome Atlas (TCGA) have been employed. The input data for the training was converted into RGB formats and the training was performed by a CNN approach.

Nirmalakumari et al. [18] focused on classifying the PCa in an accurate manner. Open-source two-class prostate data which contains 136 samples and 12,600 genes are taken into account. At first, PCA and Kruskal-Wallis test are employed to determine the informative genes. Next, they are categorized by utilizing LDA, SVM, XGB, and KNN classification to classify prostate patients as normal or abnormal. Ahn et al. [19] aimed at addressing how far the DL method could learn for recognizing cancer. They incorporated gene expression data from the GEO, TCGA, TARGET, and GTEx database including 12,842 normal gene expression data and 13,406 cancer from twenty-four distinct tissues. First, a DNN system is trained for identifying normal and cancer samples with different gene selection approach. Al-Obeidat et al. [20] introduce gene encoder, an unsupervised 2-phase FS method for the classification of cancer sample. Initially, they aggregate three filter methodologies, such as spectral-based FS, PCA, and correlation methods. Then, the GA approach is utilized that estimates the chromosome using the AE-based clustering. The resulting feature subsets are utilized for classifier process.

## 3. The Proposed Model

In this study, a new AIFSDL-PCD technique has been developed for the detection and classification of PCa. The proposed AIFSDL-PCD technique incorporates different processes, namely, preprocessing, CIWO based FS, DNN based classification, and RMSprop based hyperparameter tuning. The application of CIWO based FS technique helps for reducing the computational complexity and improving the classification accuracy.  Figure 1 illustrates the overall working process of AIFSDL-PCD technique.

### 3.1. Data Preprocessing

The presented work utilizes the preprocessed step as a huge volume of biological information has high level of noise as well as bias. So, the gene term dataset needs the subsequent more than one preprocessed step previously executing design investigation [21].

- The gene expression data demonstrate skewed distributions where lower stated genes were among zero as well as one, but the extreme term genes are among one as well as infinity. Thus, once a parametric statistical test was implemented for such asymmetric data, at the end outcome is from biased result. For overcoming this challenge, the log transformation was utilized for making the data further symmetric that is anticipated for giving an accurate outcome under statistical tests.
- The replicate of handling look at the repeated gene identify from a dataset that is afterward exchanged by its average value, so extracting the unpredictable repetitions.
- This design standardized was utilized that removes the scale variance among the features by subtracting the instance average and dividing the value by standard deviation (SD).
- The occurrence of missing value of gene term has allowed for average form.
- The flat pattern filter was utilized which removes genes for reducing the difficulty of dataset which is employed to biological significant study.

### 3.2. Design of CIWO-Based Feature Selection Technique

At this stage, the preprocessed data is passed as input to CIWO technique for the optimum selection of feature subsets. The IWO technique is stimulated by the procedure of adaptability, reproduction, and existence [22]. Accordingly, weeds represent unwanted plants which have aggressive behaviour for growth and are threats to another crop and prevent them from growing. This approach is fast, simple, and highly efficient in detecting the optimum point. Indeed, this method is depending on the natural features of weeds like struggle for existence, seed production, and growth. The description of IWO approach is given in the following:

- The evaluation of objective function and the production of arbitrary population initialization (seed distribution) from chosen domain are done, so that an initial population from the problem solving domains are distributed randomly and estimated.
- Reproduction depends on upgraded SD and competency. All the members of population, based on their capacity, yield seeds according to the maximum and minimum competence among the two predetermined quantities.

The amount of seeds that every plant could yield linearly differs in the small amount of seeds to the maximal number (*S*_min_; *S*_max_). The amount of seeds generated near every weed is defined by the following equation:

(1) $$\begin{array}{c} {\text{Seed}}_{i}=\text{Round}\left\{S_{\text{min}}+\left(S_{\max}-S_{\min}\right)\times \frac{N_{\text{weed}}-{\text{rank}}_{i}}{N_{\text{weed}}-1}\right\}, \end{array}$$

where rank_i_ represents the rank of *i* seed, Round denotes the function to iteration number, N_weed_ indicates the amount of initial weeds, *S*_max_ and *S*_min_ signify the least and most seeds which are generated near every weed, correspondingly, and Seed_i_ implies the amount of seeds generated near ith weed. The seed generated in the searching space is distributed arbitrarily in the problem space with standard distribution (predefined variance and average of zero); the seed is dispersed near to its parent (weeds). The values of SD (*r*_iter_) reduce nonlinearity in all iterations in the first value (*r*_initial_) to the last values (*r*_final_) as follows. For example, the closer we get to the end of the process, the further the seeds are produced near the answer attained and the less distributed they are than at the beginning of the process.

(2) $$\begin{array}{c} \sigma_{\text{iteri}}={\left(\frac{\text{max}\_\text{iter}-{\text{iter}}_{i}}{\text{max}\_\text{iter}}\right)}^{n}\left(\sigma_{\text{initial}}-\sigma_{\text{final}}\right)+\sigma_{\text{final}}. \end{array}$$

In equation (2), max_iter denotes the maximal amount of iterations, iter_*i*_ indicates *i*^th^ iteration, *n* represent the nonlinear coefficient, and *σ*_iter_*i*__ indicates the SD of *i*^th^ iteration. When the weed does not reproduce, it would pass away. Hence, competition among weeds is required for limiting the maximal amount. Assuming that, after many stages of iteration, the amount of seeds owing to reproduction rises, an algorithm must be determined for controlling the entire amount of them. Once the maximal amount of allowed seeds (*P*_max_) is attained, the weaker seeds must be removed; thus the seed population remains at the maximal number (*P*_max_). This procedure is repeated till the plant reaches the optimal by checking the end condition.

To improve the efficiency of the IWO algorithm, the CIWO algorithm has been derived by the integration of chaos theory. Chaos is a widespread nonlinear phenomenon by its nature and is a feature of randomness, ergodicity, sensitivity to primary states, etc. [23]. Because of the features of ergodicity and randomness, chaotic motion traverses each state from particular range based on its individual law without repetition. So, when it can be utilized with chaos variables for searching optimum, it undoubtedly has further benefits to arbitrary searches. The chaos ergodicity feature was utilized for optimizing the search and avoiding fall as to local minima; so, chaos optimized search technique developed a new optimized approach. The chaotic orders created by distinct mappings are utilized as tent map, sinusoidal map, logistic map, singer map, and sine map. Many chaotic maps are tried and an optimum one is selected for combining with IWO technique. Because of the primary testing, logistic map attained optimum outcomes. Therefore, the chaotic orders were created by utilizing logistic map as

(3) $$\begin{array}{c} x_{i+1}=ux_{i}\left(1-x_{i}\right), \end{array}$$

where *u* refers to the control parameter and assumes *u*=4. When *u*=4, the logistic mapping derives as to detailed chaotic state. Assume *x*_*i*_ ∈ (0,1) and *x*_*i*_ ≠ 0.25, 0.5, 0.75.

The preliminary weed population Seed_*i*_ is mapped to chaotic order which is created based on (3), resulting in equivalent chaotic seed population *pch*.

(4) $$\begin{array}{c} pch=x_{i}*{\text{Seed}}_{i}. \end{array}$$

During the IWO based FS process, when the feature vector size is *N*, the number of possible feature arrangements is found to be 2^*N*^, which is massive. The IWO algorithm looks for the optimal subset of features in the search space. Algorithm 1 shows the pseudocode of IWO algorithm.

The FS problem can be considered as a multiobjective issue which aims for reducing the number of chosen features and increasing the classification accuracy. Therefore, the fitness function of the IWO algorithm can determine the solutions constructed to maintain a tradeoff among two objectives.

(5) $$\begin{array}{c} \text{fitness}=\alpha \Delta_{R}\left(D\right)+\beta \frac{\left|Y\right|}{\left|T\right|}, \end{array}$$

where Δ_*R*_(*D*) denotes the error rate of the classification model, |*Y*| indicates the number of features chosen by the IWO algorithm, and |*T*|  represents the available set of features that exist in the present dataset.

### 3.3. Design of Optimal DNN-Based Classification Model

During classification process, the chosen subset of features is passed into the DNN model for PCa detection. The DNN is a version of MLP and that is kind of FFNN with two or more layers with 1 input, 1 output layer, and one or more hidden layers. All layers have many neurons and FC with neurons from forwarding direction [24]. The model is mathematically determined as *O* : ℝ^*m*^ × ℝ^*n*^. An input vector *x*=*x*_1_, *x*_2_, *x*_3_,…, *x*_*m*_ and their size is ‘*m*' and resultant vector has *O*(*x*) and their size ‘*n*'. The calculation of all hidden layers *h*_*j*_ is determined mathematically as

(6) $$\begin{array}{c} h_{j}\left(x_{j}^{l+1}\right)=f\left(Z_{ij}+b_{j}^{\left(l+1\right)}\right), \end{array}$$

(7) $$\begin{array}{c} Z_{\text{ij}}=x_{i}^{l}w_{ij}^{\left(l,l+1\right)}. \end{array}$$

Every lower layer neuron individual is linked to neuron *j*. In equations (6) and (7), *x*_*i*_^(*l*)^ has neuron *i* activation function at layer *l* and *Z*_*ij*_ refers to the influence of neuron *i* at layer *l* to activation of neuron *j* at layer *l*+1. The function *f* refers to the nonlinear activation function, *w*_*ij*_^(*l*, *l*+1)^ implies the weight, and *b*_*j*_^*l*+1^ represents the bias of neuron *j*. This technique utilizes softmax function as nonlinear activation function to multiclass classifier. In several stacking hidden layers MLP has been named DNN. Generally, the DNN with several hidden layers is expressed as

(8) $$\begin{array}{c} H_{l}\left(x\right)=H_{l}\left(H_{l-1}\left(H_{l-2}\left(\ldots \left(H_{1}\left(x\right)\right)\right)\right)\right). \end{array}$$

The DNN framework has 2 hidden layers. It gets inputs *x*=*x*_1_, *x*_2_, *x*_3_,…, *x*_*m*_ and outputs were *o*=*o*_1_, *o*_2_,…, *o*_*c*−1_, *o*_*c*_. Figure 2 showcases the framework of DNN.

Further advanced typical feedforward network DNN can be utilized with all the hidden layers having ReLU nonlinear activation functions. It is used for decreasing the state of vanishing and error gradient problems [24] and is related to another nonlinear activation function ReLU which is quicker and simpler for training the technique with huge hidden layer.

The loss function has optimum parameters that can be vital for achieving higher efficiency. The target and forecast values variance was computed as utilizing loss function. It could be defined as

(9) $$\begin{array}{c} d\left(t,p\right)={\left\|t-p\right\|}_{2}^{2}. \end{array}$$

It attempts for learning an estimate to identify the function, with the learning procedure explained as minimizing reform error as illustrated in equation (9), where *t* and *p* refer to the target as well as forecasted values correspondingly. The loss function is used for identifying that forecasted value diverges in the target value. The target is fed to model along with features for calculating the loss function and classifying the attack. The negative log probability with *t* and probability distribution *p*(*p* *d*) are utilized to target and forecast classes correspondingly from multiclass classifier. It could be written as

(10) $$\begin{array}{c} d\left(t,p\left(p,\;d\right)\right)=-\log\;p{\left(p\;d\right)}_{t}. \end{array}$$

To effectually tune the hyperparameters of the DNN model, the RMSprop optimizer is utilized. RMSprop is the enhancement form of Adagrad; the upgrade procedure of RMSprop is the same as Adagrad [25]. For RMSprop, an exponentially decaying average of squared gradient is computed initially.

(11) $$\begin{array}{c} G_{t}=\beta G_{t-1}+\left(1-\beta \right)g_{t}⊙g_{t}\\ =\left(1-\beta \right)\sum_{\tau =1}^{t}\beta^{t-\tau }g_{\tau }⊙g_{\tau }, \end{array}$$

where *β* refers to the decay rate that is generally offered which is fixed to 0.9. And the upgrade value of parameters from RMSprop is similar to Adagrad:

(12) $$\begin{array}{c} △\theta_{t}=-\frac{\alpha }{\sqrt{G_{t}+\varepsilon }}⊙g_{\tau }. \end{array}$$

Also, the simplified concept of Adagrad technique is implemented. *g*_*t*_′ is explained as

(13) $$\begin{array}{c} g_{t}^{\prime }=\frac{1}{\sqrt{G_{t}+\varepsilon }}⊙g_{\tau }, \end{array}$$

and the upgrade value of RMSprop has been determined as

(14) $$\begin{array}{c} \Delta \theta_{t}=-\alpha g_{t}^{\prime }. \end{array}$$

So, the RMSprop is an optimized technique dependent upon gradient actually. To provide analysis, the rate of learning optimized technique was utilized for improving the trained efficiency.

## 4. Results and Discussion

The performance validation of the AIFSDL-PCD technique takes place using an open access dataset, including 102 tissue instances (52 prostate tumors and 50 normal tissues) with 2135 genes. The proposed model is simulated using Python 3.6.5 tool.  Table 1 and Figure 3 illustrate the result analysis of the optimal DNN model under ten iterations. The results exhibited that the optimal DNN algorithm has accomplished satisfactory outcomes. For instance, under iteration 1, the optimal DNN model has provided sens_*y*_, spec_*y*_, prec_*n*_, accu_*y*_, and *F*_score_ of 96.30%, 95.56%, 96.67%, 96.64%, and 96.32%, respectively.

In line with this, under iteration 4, the optimal DNN method has provided sens_*y*_, spec_*y*_, prec_*n*_, accu_*y*_, and *F*_score_ of 96.13%, 96.34%, 96.15%, 96.19%, and 96.19% correspondingly. Meanwhile, under iteration 6, the optimal DNN approach has offered sens_*y*_, spec_*y*_, prec_*n*_, accu_*y*_, and *F*_score_ of 95.59%, 95.63%, 96.55%, 95.86%, and 95.53%, respectively. Eventually, under iteration 8, the optimal DNN technique has showed sens_*y*_, spec_*y*_, prec_*n*_, accu_*y*_, and *F*_score_ of 95.56%, 96.88%, 96.34%, 95.72%, and 96.43% correspondingly. At last, under iteration 10, the optimal DNN methodology has provided sens_*y*_, spec_*y*_, prec_*n*_, accu_*y*_, and *F*_score_ of 96.44%, 96.18%, 96.15%, 96.38%, and 96.05% correspondingly.

The ROC analysis of the optimal DNN approach is implemented in Figure 4. The figure displayed that the optimal DNN approach has accomplished optimum ROC classification performance with the increased ROC of 99.3002.

Table 2 and Figure 5 showcase the result analysis of the AIFSDL-PCD approach under ten iterations. The outcomes showed that the AIFSDL-PCD technique has accomplished satisfactory outcomes. For instance, under iteration 1, the AIFSDL-PCD algorithm has provided sens_*y*_, spec_*y*_, prec_*n*_, accu_*y*_, and *F*_score_ of 97.75%, 97.26%, 96.87%, 97.47%, and 97.58% correspondingly. Likewise, under iteration 4, the AIFSDL-PCD technique has given sens_*y*_, spec_*y*_, prec_*n*_, accu_*y*_, and *F*_score_ of 97.49%, 97.10%, 96.92%, 97.18%, and 97.07% correspondingly. In the meantime, under iteration 6, the AIFSDL-PCD model has provided sens_*y*_, spec_*y*_, prec_*n*_, accu_*y*_, and *F*_score_ of 97.43%, 96.92%, 97.39%, 97.27%, and 96.89%, respectively. Eventually, under iteration 8, the AIFSDL-PCD approach has offered sens_*y*_, spec_*y*_, prec_*n*_, accu_*y*_, and *F*_score_ of 97.18%, 97.37%, 97.34%, 97.06%, and 97.75% correspondingly. At last, under iteration 10, the AIFSDL-PCD model has provided sens_*y*_, spec_*y*_, prec_*n*_, accu_*y*_, and *F*_score_ of 97.28%, 97.66%, 97.23%, 97.28%, and 96.51% correspondingly.

The ROC analysis of the AIFSDL-PCD technique is performed in Figure 6. The figure exhibited that the AIFSDL-PCD technique has accomplished better ROC classification performance with a maximum ROC of 99.6769.

Figure 7 demonstrates the accuracy analysis of AIFSDL-PCD technique on the test dataset. The outcomes exhibited that the AIFSDL-PCD system has accomplished increased performance with improved training and validation accuracy. It can be clear that the AIFSDL-PCD methodology has reached enhanced validation accuracy on the training accuracy.

Figure 8 depicts the loss analysis of the AIFSDL-PCD approach on the test dataset. The outcomes recognized that the AIFSDL-PCD methodology has resulted in a proficient outcome with lesser training and validation loss. It can be obvious that the AIFSDL-PCD algorithm has obtainable lesser validation loss on the training loss.

To portray the better classification performance of the AIFSDL-PCD method, a comparative *acc*_*y*_ analysis is made in Table 3 and Figure 9 [26, 27]. The results show that the GA-KNN + SVM model has failed to achieve proficient classification performance. At the same time, the PLR-MC, RFLD-MC, and Bio-HEL techniques have accomplished moderately closer accuracy values. Along with that, the CSF-RC and optimal DNN techniques have managed to demonstrate reasonable accuracy values. However, the AIFSDL-PCD technique has resulted in superior performance with higher accuracy of 0.9719. From the aforementioned tables and figures, it can be obvious that the AIFSDL-PCD method is found to be an effective tool for PCa detection and classification.

## 5. Conclusion

In this study, a new AIFSDL-PCD method has been developed for the detection and classification of PCa. The proposed AIFSDL-PCD technique incorporates different processes, namely, preprocessing, CIWO based FS, DNN based classification, and RMSprop based hyperparameter tuning. The application of CIWO based FS technique helps for reducing the computational complexity and improves the classification accuracy. For examining the betterment of the AIFSDL-PCD technique, a comprehensive experimental analysis is carried out and the results are examined under several aspects. The experimental results reported the supremacy of the AIFSDL-PCD technique over the other techniques in terms of different measures. Therefore, the AIFSDL-PCD technique can be applied as a proficient tool for the detection and classification of PCa. As a part of future extension, hybrid DL based classifiers with metaheuristics based hyperparameter optimizers can be developed to boost the PCa detection results.

## Figures and Tables

**Figure 1:** Overall process of AIFSDL-PCD technique.

**Figure 2:** DNN structure.

**Figure 3:** Result analysis of optimal DNN technique.

**Figure 4:** ROC analysis of optimal DNN technique.

**Figure 5:** Result analysis of AIFSDL-PCD approach.

**Figure 6:** ROC analysis of AIFSDL-PCD technique.

**Figure 7:** Accuracy graph analysis of AIFSDL-PCD technique.

**Figure 8:** Loss graph analysis of AIFSDL-PCD technique.

**Figure 9:** Accuracy analysis of AIFSDL-PCD technique with existing manners.

**Algorithm 1:** Pseudocode of IWO algorithm.

**Table 1:** Result analysis of optimal DNN model

No. of iterations	Sensitivity	Specificity	Precision	Accuracy	*F*-score
Iteration 1	96.30	95.56	96.67	96.64	96.32
Iteration 2	96.20	96.46	96.57	96.50	96.97
Iteration 3	95.82	96.64	96.55	95.99	95.95
Iteration 4	96.13	96.34	96.15	96.19	96.19
Iteration 5	96.25	95.66	96.75	96.51	95.63
Iteration 6	95.59	95.63	96.55	95.86	95.53
Iteration 7	95.92	96.04	96.11	95.99	96.04
Iteration 8	95.56	96.88	96.34	95.72	96.43
Iteration 9	96.17	95.57	96.53	96.31	96.27
Iteration 10	96.44	96.18	96.15	96.38	96.05
Average	**96.04**	**96.10**	**96.44**	**96.21**	**96.14**

**Table 2:** Result analysis of proposed AIFSDL-PCD model.

No. of iterations	Sensitivity	Specificity	Precision	Accuracy	*F*-score
Iteration 1	97.75	97.26	96.87	97.47	97.58
Iteration 2	97.25	97.30	96.69	96.83	97.48
Iteration 3	97.59	97.21	97.34	97.41	97.06
Iteration 4	97.49	97.10	96.92	97.18	97.07
Iteration 5	97.11	96.60	96.90	96.69	97.22
Iteration 6	97.43	96.92	97.39	97.27	96.89
Iteration 7	96.87	97.27	97.34	97.06	97.75
Iteration 8	97.18	97.37	97.43	97.34	97.71
Iteration 9	96.51	97.78	97.25	97.41	97.51
Iteration 10	97.28	97.66	97.23	97.28	96.51
**Average**	**97.25**	**97.25**	**97.14**	**97.19**	**97.28**

**Table 3:** Comparative analysis of AIFSDL-PCD approach with existing techniques.

Methods	Accuracy
PLR-MC	0.9460
RFLD-MC	0.9340
Bio-HEL	0.9400
SVM model	0.9120
GA-KNN + SVM	0.8571
CSF-RC	0.9510
Optimal DNN	0.9621
AIFSDL-PCD	0.9719

## Data Availability

Data sharing is not applicable to this article as no datasets were generated during the current study.
